# Association of Chest Anteroposterior Radiography with Computed Tomography in Patients with Blunt Chest Trauma

**DOI:** 10.1155/2023/6678211

**Published:** 2023-06-06

**Authors:** Young Un Choi, Chang Whan Kim, JiHye Lim, Il Hwan Park, Chun Sung Byun

**Affiliations:** ^1^Department of Trauma Surgery, Yonsei University, Wonju College of Medicine, Wonju, Republic of Korea; ^2^Department of Cardiovascular and Thoracic Surgery, Yonsei University, Wonju College of Medicine, Wonju, Republic of Korea; ^3^National Health Big Data Clinical Research Institute, Yonsei University, Wonju College of Medicine, Wonju, Republic of Korea

## Abstract

**Background:**

In cases of chest trauma, computed tomography (CT) can be used alongside chest anteroposterior (AP) radiography and physical examination during initial evaluation. Performing a CT scan may be difficult if a patient has unstable vital signs. In contrast, radiography may not always reliably diagnose nonmarked pneumothorax or extensive subcutaneous emphysema.

**Objectives:**

This study aimed to determine the agreement between chest radiography and CT findings in patients with blunt chest trauma. The study also aimed to determine the occurrence of occult pneumothorax and clarify the proportion of subcutaneous emphysema and pneumothorax detected through radiography and CT, respectively.

**Methods:**

We included patients (*n* = 1284) with chest trauma who were admitted to the emergency room of a tertiary hospital between January 2015 and June 2022. We excluded patients aged <18 years, those with stab injury, those without radiography and CT findings, and patients who required iatrogenic intervention, such as chest tube insertion, before imaging. We recorded age, sex, trauma mechanism, and Abbreviated Injury Scale score for each patient. From radiography and CT scans, we recorded the presence of rib fracture, subcutaneous emphysema, lung contusion, pneumothorax, and pneumomediastinum. The accuracy, sensitivity, specificity, and positive and negative predictive values were calculated to assess the reliability of radiography as a predictor of CT-based diagnosis.

**Results:**

Radiography exhibited a specificity of nearly 100% for all items. In most cases, findings that could not be confirmed by CT were not evident on radiographs. The incidence of occult pneumothorax was 87.3%. When subcutaneous emphysema was observed on radiography, CT findings indicated pneumothorax in 96.7% of cases.

**Conclusions:**

In situations where the patient's vital signs are unstable and performing a CT scan is not feasible, the presence of subcutaneous emphysema on radiography may indicate the need for chest decompression, even if pneumothorax is not observed.

## 1. Introduction

According to the Statistical Yearbook (the Korean Trauma Database) of the trauma registration system issued by the National Medical Center in 2021, severe trauma frequently affects the chest after the head and neck [1]. During the initial assessment of trauma patients, various methods such as physical examination, anteroposterior (AP) radiography, and extended focused assessment using sonography in trauma (eFAST) can all be used to evaluate the chest [2]. Once the vital signs stabilize, a secondary assessment with chest computed tomography (CT) can be performed to accurately assess the degree of damage to the chest. However, if the vital signs are unstable, CT cannot immediately be performed, and the Advanced Trauma Life Support guidelines state that the degree of damage should be assessed as accurately as possible at initial examination without CT. Nonetheless, severe subcutaneous emphysema may hinder the effectiveness of eFAST due to the air layer obstructing auscultation. Additionally, nonmarked pneumothorax may not easily be detected on an AP radiograph because of overlapping lung structures [3]. Even in the case of rib fractures, it may be difficult to detect fine fractures in the posterior or lateral portion of the chest with radiographs due to overlapping structures.

Figure 1 illustrates occult pneumothorax on radiography and CT. Mild pneumothorax cannot be observed on a radiograph taken in the supine position because of overlapping structures.

Thus, this study aimed to determine the agreement between chest AP radiographic and CT findings in patients with blunt chest trauma. Specifically, we aimed to establish the prevalence of occult pneumothorax and the respective proportion of emphysema and pneumothorax findings on radiography and CT.

## 2. Materials and Methods

The study included patients with chest trauma who were transferred to the emergency department of the hospital between January 2015 and June 2022. We excluded patients who were <18 years, those with stab injury, those with no radiography and CT data, or patients who underwent iatrogenic intervention, such as chest tube insertion before imaging examinations. A total of 1836 patients were included, 551 patients were excluded, resulting in 1284 patients studied. Medical records were retrospectively analyzed and the following data were extracted: age, sex, Injury Severity Score (ISS), chest Abbreviated Injury Scale (AIS) score, and trauma mechanisms. From radiographs and CT images, we recorded the presence or absence of rib fracture, subcutaneous emphysema, lung contusion, pneumothorax, and pneumomediastinum. All the images were assessed by a radiologist and a chest surgeon. The study was approved by the institutional review board (IRB no. CR 323016).

### 2.1. Statistical Analysis

Continuous variables were tested for normality using the Shapiro–Wilk test, and no variables followed a normal distribution. Thus, continuous data are reported as medians (interquartile ranges). Categorical variables are reported as frequencies (percentages). The accuracy, sensitivity, specificity, and positive and negative predictive values were calculated to assess the reliability of radiography as a predictor of the CT-based diagnosis. All statistical analyses were performed using the SAS statistical software (version 9.4; SAS Institute, Cary, North Carolina, US) and R version 4.2.1 (R Core Team, Vienna, Austria).

## 3. Results

The average age of the patients was 59 years, and most of them were male (75.3%). The average ISS was 17, the chest AIS score was 3 for most mechanisms, and traffic accidents and falls were the most common mechanisms of injury (Table 1).

The sensitivity of radiography compared to CT was high for rib fractures (72.8%). For all diagnostic items, the specificity of radiography, which is the predicted value for CT, was nearly 100%.

In most cases, findings that could not be confirmed on CT were not evident on radiographs. CT scan was able to confirm the findings yielded by radiography in almost all cases. These findings indicate the reliability of the readings (Table 2). The incidence of occult pneumothorax was 53.43% (686/1284 cases). The proportion of cases in which radiographic and CT diagnoses were completely consistent in all four items was 13.94% (*n* = 179).

Table 3 presents CT findings with respect to positive radiography findings. Rib fractures on radiography were associated with lung contusions on CT in 90.7% of cases. Lung contusions on radiography were associated with rib fractures on CT in 95.2% of cases. The most important finding on radiography was subcutaneous emphysema, which was associated with pneumothorax on CT in 96.7% of cases. Thus, subcutaneous emphysema observed on radiography may be a diagnostic marker for pneumothorax clinical practice. More than 90% of the CT scans with rib fractures and contusions were positive for pneumothorax on radiography.

## 4. Discussion

Occult pneumothorax refers to pneumothorax that is observed on CT but not on plain radiography [4], and it may directly impact a patient's survival. Occult pneumothorax does not always require intervention and is often treated conservatively [5]. However, if missed, it can progress to tension pneumothorax, which is more likely to develop when a ventilator is required [6]. Occult pneumothorax has an incidence of 8–15% in trauma patients [7–9]. As confirmed in our study, it has a fairly high frequency of 53.43% in patients with blunt chest trauma, and if not recognized timeously, resuscitation techniques, such as intubation in patients with reduced consciousness, may result in tension pneumothorax and obstructive shock [6]. Therefore, the prompt diagnosis of occult pneumothorax is crucial, and repeated physical examinations and eFAST can help in this regard. Many studies have reported radiographic findings suggesting occult pneumothorax [10–14].

Our study also considered whether additional factors evident on radiographs could predict occult pneumothorax. We found that emphysema observed on chest AP radiographs indicates damage to the parietal pleura of the thorax; therefore, its presence may indicate pneumothorax. In our study, pneumothorax was confirmed via CT in 96.7% of patients with subcutaneous emphysema on radiography. Thus, subcutaneous emphysema observed on radiographs may be a stronger indicator of pneumothorax than rib fractures or lung contusions evidenced on using this imaging modality.

### 4.1. Limitations

In this study, the presence or absence of the disease was confirmed, but we did not report the extent or location of the trauma. Therefore, even if radiography and CT reported identical diagnostic names, the injuries could have occurred at different locations, and the degree of fracture, contusion, and pneumothorax cannot be distinguished. In occult pneumothorax, many cases are not clinically significant if the extent of pneumothorax is small, and cases where pneumothorax is not visible on radiography are commonly followed up without chest tube insertion. In many cases, not all parts of the chest can be imaged during chest AP radiography, and the sensitivity of radiography to rib fractures and subcutaneous emphysema may be reduced.

## 5. Conclusions

Microfractures, fractures of the posterior chest, and microscopic pneumothorax are not visible on chest AP radiography but may be confirmed using CT, which is better able to identify chest trauma than chest AP radiography. In particular, simple trauma-related pneumothorax should be detected timeously because it can develop into tension pneumothorax in situations when intubation is required. Subcutaneous emphysema on a chest AP radiograph may be suggestive of pneumothorax. Clinically, subcutaneous emphysema as revealed by AP radiographs may indicate the need for chest decompression; this is particularly important when a patient's vital signs are unstable and CT cannot be performed.

## Figures and Tables

**Figure 1:** Imaging findings of a 48-year-old male traffic accident patient. (a) Lung contusion can be seen on the chest anteroposterior (AP) radiograph. (b) Lung contusion and pneumothorax can be seen on the chest computed tomography image. Pneumothorax was not visible in the chest AP radiograph.

**Table 1:** Basic characteristics of the patients.

Variables	Total (*n* = 1284)	Traffic accident (*n* = 687)	Fall (*n* = 344)	Slip (*n* = 77)	Crush injury (*n* = 26)	Assault (*n* = 126)	Explosion injury (*n* = 2)	Drowning (*n* = 1)	Other (*n* = 21)
*Injury mechanism*									
Age (years)	59.0 (50.0–68.5)	60.0 (49.0–70.0)	58.5 (50.0–64.0)	67.0 (55.0–78.0)	65.0 (51.0–73.0)	58.0 (48.0–66.0)	42.5 (42.0–43.0)	38.0 (38.0–38.0)	62.0 (56.0–80.0)
Sex (male)	967 (75.3)	488 (71.0)	285 (82.9)	50 (64.9)	26 (100.0)	100 (79.4)	2 (100.0)	1 (100.0)	15 (71.4)
ISS	17.0 (13.0–22.0)	18.0 (13.0–25.0)	17.0 (13.0–24.0)	9.0 (9.0–10.0)	17.0 (13.0–25.0)	13.0 (9.0–18.0)	32.5 (8.0–57.0)	8.0 (8.0–8.0)	22.0 (17.0–26.0)
Chest AIS score	3 (3.0–3.0)	3.0 (3.0–3.0)	3.0 (3.0–3.0)	3.0 (3.0–3.0)	3.0 (3.0–3.0)	3.0 (3.0–3.0)	3.0 (2.0–4.0)	2.0 (2.0–2.0)	3.0 (3.0–3.0)

*Blunt or burn*									
Blunt	1282 (99.8%)	687 (100.0%)	344 (100.0%)	77 (100.0%)	26 (100.0%)	126 (100.0%)	0 (0.0%)	1 (100.0%)	21 (100.0%)
Burn	2 (0.2%)	0 (0.0%)	0 (0.0%)	0 (0.0%)	0 (0.0%)	0 (0.0%)	2 (100.0%)	0 (0.0%)	0 (0.0%)

Values are presented as median (interquartile range) or *n* (%). ISS: injury severity score; AIS: Abbreviated Injury Scale.

**Table 2:** Statistics of positive findings on radiography when the computed tomography scan finding is positive.

	Accuracy (%)	Sensitivity (%)	Specificity (%)	PPV (%)	NPV (%)	*F* score (%)	Kappa coefficient
Rib fracture	74.9	72.8	100	100	23.5%	84.3	0.292
Lung contusion	50.5	43.8	99.4	99.8	19.4%	60.9	0.155
Subcutaneous emphysema	83.5	56.0	99.9	99.6	79.2	71.7%	0.613
Pneumothorax	46.7	12.7	100.0	100.0	42.1	22.6%	0.102

PPV, positive predictive value; NPV, negative predictive value.

**Table 3:** Computed tomography findings in relation to positive radiography findings.

Radiography	CT rib fracture		CT contusion		CT subcutaneous emphysema		CT pneumothorax	
	Negative	Positive	Negative	Positive	Negative	Positive	Negative	Positive
Rib fracture	0 (0.0)	863 (100.0)	80 (9.3)	783 (90.7)	455 (52.7)	408 (47.3)	295 (34.2)	568 (65.8)
Lung contusion	24 (4.8)	472 (95.2)	1 (0.2)	495 (99.8)	257 (51.8)	239 (48.2)	152 (30.7)	344 (69.34)
Subcutaneous emphysema	0 (0.0)	270 (100.0)	11 (4.1)	259 (95.9)	1 (0.4)	269 (99.6)	9 (3.3)	261 (96.7)
Pneumothorax	10 (10.0)	90 (90.0)	3 (3.0)	97 (97.0)	40 (40.0)	60 (60.0)	0 (0.0)	100 (100.0)

## Data Availability

The datasets used and/or analyzed in the current study are available from the corresponding author upon reasonable request.
